The article "Antiarthritic Activity of Qi-Wu Rheumatism Granule (a Chinese Herbal Compound) on Complete Freund's Adjuvant-Induced Arthritis in Rats" was retracted in 2026. Reasons: plagiarized images; overlap with other authors' work; unreliable results or conclusions; concerns about the images.

# Antiarthritic Activity of Qi-Wu Rheumatism Granule (a Chinese Herbal Compound) on Complete Freund's Adjuvant-Induced Arthritis in Rats

**DOI:** 10.1155/2017/1960517

**Published:** 2017-11-07

**Authors:** Qi Xu, Yong Zhou, Rong Zhang, Zhan Sun, Lu-feng Cheng

**Affiliations:** ^1^Department of Immunology, School of Preclinical Medicine, Xinjiang Medical University, Urumqi 830011, China; ^2^Department of Biology, School of Preclinical Medicine, Xinjiang Medical University, Urumqi 830011, China; ^3^Center of Functional Experiment, School of Preclinical Medicine, Xinjiang Medical University, Urumqi 830011, China; ^4^Department of Pharmacology, School of Preclinical Medicine, Xinjiang Medical University, Urumqi 830011, China

## Abstract

**Objective:**

The aim was to study the therapeutic effects and mechanisms of QWRG on adjuvant-induced RA in rats.

**Methods:**

The RA rat models were manipulated and subsequently divided into five experimental groups: AIA, DEX, and QWRG groups. The paw volume, body weight, arthritic score, and mechanical nociceptive threshold were assessed. The serum levels of the RF, MDA, ALP, AST, ALT, IL-1*β*, IL-2, IL-16, and TNF-*α* were measured. The proliferative capacity of lymphocytes was evaluated, and the synovial tissue was histopathologically examined.

**Results:**

The paw swelling and arthritic scores were relieved, and the variation of relative body weight and mechanical nociceptive threshold had improved in the AIA rats. The serum levels of RF, MDA, ALP, AST, and ALT were alleviated, and the inflammation and cartilage damage were effectively attenuated in the AIA rats. Simultaneously, the inflammation of the synovial cavity was alleviated, and the grading of synovitis reduced by inhibiting the expressions of IL-1*β*, TNF-*α*, and IL-16 in the serum and synovium tissue.

**Conclusion:**

Our results suggested that the antiarthritic properties of QWRG may be due to immunodepression and downregulation of inflammatory cytokines, which may be a potential candidate for the treatment of RA.

## 1. Introduction

Rheumatoid arthritis (RA) is an autoimmune disease characterized by chronic, symmetric, inflammatory, and systemic manifestations and affects between 0.3 and 1% of the population worldwide [1]. The disease appears in most cases between 50 and 60 years of age and women are more affected than men [2, 3]. In patients with RA, a joint deformation is observed with an increase in the extent of loss of function and cartilage and bone destruction [4]. In terms of the characteristics of the disease, RA shows stages of pathological process, and early symptoms of heat, swelling, pain, and decreased joint function; the late stage shows different degrees of joint stiffness and deformity accompanying bone damage and disability risk [5]. With the development of RA, it characteristically affects the small joints of the hands and feet resulting in a gradual painful swelling, exaggerated, and abnormal development of the synovium, pannus formation, and changes in the morphology of the joint [6]. Although the pathogenesis and mechanisms of RA are not fully understood, it is stated that part of the RA pathogenesis is the retention of microbial products in the synovial tissue and persistent infection of the joint articular surface, which induces an immune reaction, ultimately altering the integrity of these joint components.

The article "Antiarthritic Activity of Qi-Wu Rheumatism Granule (a Chinese Herbal Compound) on Complete Freund's Adjuvant-Induced Arthritis in Rats" was retracted in 2026. Reasons: plagiarized images; overlap with other authors' work; unreliable results or conclusions; concerns about the images.

Currently, there is no effective cure for RA [7]. Although many current therapies including nonsteroidal anti-inflammatory drugs, glucocorticosteroids, and biological agents improve pain, fatigue, and disability, they mainly focus on controlling synovitis. Furthermore, long-term, large-dose administrations of these agents could lead to relative limited effectiveness and severe negative side effects [8, 9]. In addition, therapeutic effects in RA might be achieved by antagonizing these proinflammatory mediators. Newer therapies such as antitumor necrosis factor- (TNF-) *α* therapy, anti-CD20 therapy, and CD80/86 blockade are required to inhibit the underlying immune process. However, all these antirheumatic drugs are associated with numerous side effects coupled with lengthy treatment duration and potential unknown threats [10–12]. Consequently, it has become an inevitable trend to identify an effective anti-RA drug with high therapeutic effects and fewer side effects. The search for traditional herbal drugs that are more effective, safer, and economical has attracted a great attention, since 80% of the world population mainly rely on herbal drugs [13]. With the long history of traditional Chinese medicine (TCM) in the treatment of RA, RA is included in the theory of TCM “arthralgia” category. The TCM treatments focus on reinforcing qi and nourishing the blood, dispelling cold and removing dampness, promoting blood circulation, dispelling wind and relieving pain, and addressing both the symptoms and root cause and strengthening the body resistance to eliminate pathogenic factors. TCM not only has the advantages of fewer side effects and lower costs but can also be used for individual treatment with multiway, multilink, multitarget effects and integral regulation [14]. It is confirmed that TCM treatment on RA could significantly improve the living quality of patients, which provides a new way to overcome many difficulties [15, 16].

Qi-Wu Rheumatism Granule (QWRG), a herbal formulation consisting of five crude drugs, namely,* milkvetch root, Radix Aconiti Preparata, scorpion, centipede, *and* geosaurus* (w : w), is considered an integral part of TCM and widely used in* Affiliated Traditional Chinese Medical Hospital of Xinjiang Medical University*. QWRG is effective for cold resistance with “antiarthromyodynia” [17], which has been long used as a folk medicine to treat RA. In RA, QWRG exerts an analgesic, anti-inflammatory, and antipyretic effect and improves the joint function. Our previous research also demonstrated that QWRG possessed a substantial anti-arthritic activity.

The article "Antiarthritic Activity of Qi-Wu Rheumatism Granule (a Chinese Herbal Compound) on Complete Freund's Adjuvant-Induced Arthritis in Rats" was retracted in 2026. Reasons: plagiarized images; overlap with other authors' work; unreliable results or conclusions; concerns about the images.

In this study, a rat model of adjuvant-induced arthritis (AIA) was established to investigate the potential therapeutic effects and mechanism of QWRG, which reflects a number of clinical characteristics of RA in humans [18, 19]. First, the safety of QWRG was evaluated in mice. Subsequently, in order to provide an effective experimental basis, and to lay a theoretical foundation for the development of new drugs for the treatment of RA with QWRG, the therapeutic effects of QWRG were evaluated in AIA rats. For this reason, the pathological change of serum biochemical indicators, immune indicators, spleen index, spleen lymphocyte proliferation, synovial membrane, and synovium expression of interleukin 1*β* (IL-1*β*), IL-2, IL-16, and tumor necrosis factor *α* (TNF-*α*) were analyzed.

## 2. Materials and Methods

### 2.1. Animals

Twenty SPF Kunming mice weighing 18–22 g (10 males and 10 females) were purchased from the Xinjiang Uygur Autonomous Region Animal Research Center (license number SCXK [Xin] 2011-0003). Sixty male Wistar rats (160 ± 20 g) were purchased from the Animal Center of Xinjiang Medical University (license number 65000700000087). All animals were provided food and water ad libitum and were maintained in a room at a controlled temperature (23–25°C) and humidity (40–50%) and under a 12/12 h light/dark cycle. The mice were allowed 7 days to adapt to the laboratory environment before the experiments. The experiments were approved by the Animal Ethical Council of Xinjiang Medical University.

### 2.2. Preparation of the QWRG Extract

The laboratory QWRG consisted of a mixture of five fruits, namely the* milkvetch root, Radix Aconiti Preparata, scorpion, centipede, *and* geosaurus* (Kangmei Pharmaceutical Co., Ltd.) in the ratio of 1 : 1 : 1 : 1 : 1 (w : w). The fruit pieces were broken and soaked in water for 12 h, decocted and boiled for 60 min, and finally gauze filtered and decocted for 30 min with another 8-fold water. Subsequently, the water filtrates were combined and heat-concentrated to a thick paste. The water filtrate was concentrated under reduced pressure at 55°C by a vacuum rotary evaporator (RE-52A, Shanghai Yarong, China) and further dried in a vacuum drying oven (DZF-6090, Shanghai Jinghong, China) to yield a solid QWRG extract at 8.6%. The dried QWRG extract was freshly prepared with normal saline before each experiment. The clinical dosage of QWRG was 124.5 g of crude extract. The water extraction content corresponded to 1 g, equivalent to 4.12 g crude drug. All other reagents used were standard laboratory reagents of analytical grade and were purchased locally.

The article "Antiarthritic Activity of Qi-Wu Rheumatism Granule (a Chinese Herbal Compound) on Complete Freund's Adjuvant-Induced Arthritis in Rats" was retracted in 2026. Reasons: plagiarized images; overlap with other authors' work; unreliable results or conclusions; concerns about the images.

### 2.3. Safety Evaluation of QWRG

After fasting for 16 h, 20 SPF Kunming mice were randomly divided into the control and QWRG group and were treated by intragastric administration with normal saline (control; 40 mL/kg) or QWRG (1.43 g/mL), respectively. Subsequently, the behavior, performance, characteristics, toxic reaction time, recovery time, and death rate were recorded before and after the treatment. Subsequently, the animals were weighed on the day of the treatment (day 0) and on days 4, 7, 10, and 14 after the treatment.

### 2.4. AIA Rats Model and Experimental Design

Male Wistar rats weighting 140–180 g were randomly divided into a normal group (10 rats) and an AIA group (50 rats). Complete Freund's Adjuvant (CFA) was obtained by mixing 7 mg/mL* mycobacterium* cheese (Lot. 0260570, Difco Int, USA), which has an efficacy 3-fold higher than that of the* Mycobacterium tuberculosis*, with the incomplete Freund's Adjuvant (Sigma, Inc., WA, USA). Rats in the AIA group were administered with a single intradermal injection of 0.1 mL CFA into the right hind paw to induce arthritis [20], while the equivalent volume of normal saline was injected to the rat in the normal group. After 7 days of inflammation, the volume of paw swelling was detected by using the Volumetric Meter (Chengdu Taimen Company, China). Subsequently, the rats were randomly divided into five experimental groups (*n* = 10 each) based on the paw swelling volume: control group, dexamethasone group (5.0 mg/kg, intraperitoneal), low QWRG group (1.0 g/kg, gavage), medium QWRG group (2.0 g/kg, gavage), and high QWRG group (4.0 g/kg, gavage). All treatments were administered orally 30 min before the CFA induction (day 0) and daily thereafter up through 35 days. Periodically, the development of arthritis was monitored by measuring the paw thickness. On day 35, at the end of the experimental period, the animals were killed by euthanasia and the blood was collected for various biochemical estimations. The spleen was immediately dissected and homogenized in ice-cold Tris HCl buffer (0.01 mol/L, pH 7.4).

### 2.5. Evaluation of AIA Development

Measurements of the paw volume, arthritic score, mechanical nociceptive threshold, thermal hyperalgesia, and body weight were recorded on days 0, 7, 14, 21, 28, and 35. The paw swelling was calculated using the following equation: paw swelling degree = (paw swelling volume)_after_  − (paw swelling volume)_before_. Randall Selitto analgesiometer (UGO Basile) was used to measure the mechanical pain threshold [20]. For each animal, the change of body weight and paw withdrawal latency responses (pain threshold) were expressed as % values relative to the preadministration value (100%) [21]. The severity of arthritis was assessed by three independent observers by visual observation. The rats were observed periodically for the severity of joint inflammation every 7 days. The severity of arthritis was graded on a five-point scale [19], with* 4* indicating edema and erythema from the ankle to the entire leg,* 3* indicating moderate edema and erythema from the ankle to the tarsal bone,* 2* indicating slight edema and erythema from the ankle to the tarsal bone,* 1* indicating slight edema and limited erythema, and* 0* indicating no edema or swelling. The arthritis score for each mouse was the sum of the severity in all the right paw (maximum four points for individual rats).

The article "Antiarthritic Activity of Qi-Wu Rheumatism Granule (a Chinese Herbal Compound) on Complete Freund's Adjuvant-Induced Arthritis in Rats" was retracted in 2026. Reasons: plagiarized images; overlap with other authors' work; unreliable results or conclusions; concerns about the images.

### 2.6. Serum Biochemical Indicators and Immune Indicators

Blood was collected from the inferior vena cava of rats in all experimental groups without anticoagulant and was centrifuged at 3,000 rpm, 4°C for 10 min at day 35 after treatments. The serum was separated and divided into aliquots at 4°C. The serum levels of the arthritis factor (RF), malondialdehyde (MDA), alkaline phosphatase (ALP), amino transaminase (AST), and alanine amino transaminase (ALT) were investigated by commercially available colorimetric assay kits (Jian Cheng Bioengineering Institute, China) according to the manufacturer's instructions. Furthermore, the serum levels of inflammation-related cytokines (IL-1*β*, TNF-*α*, IL-16, and IL-2) were evaluated using enzyme-linked immunosorbent assay (ELISA) according to the manufacturer's instructions (Bender MedSystem, Vienna, Austria). Briefly, a biotinylated antibody reagent was added to the 96-well plates, which were then filled with the homogenized serum and incubated at 37°C in CO_2_ for 2 h. After washing with phosphate-buffered saline (PBS), streptavidin-horseradish peroxidase (HRP) solution was added and the plates were incubated for 30 min at room temperature. The absorbance was measured at 450 nm using a microplate reader (iMark; Bio-Rad, Hercules, CA, USA).

### 2.7. Lymphocyte Proliferation and Spleen Index

The lymphocyte proliferation was evaluated in all rats by using the methyl thiazolyl tetrazolium (MTT) assay. Briefly, the spleen cell suspension was cultured in RPMI1640 medium, and the cell concentration was subsequently adjusted to 5 × 10^5^/mL. Subsequently, 100 *μ*L of cells was added in each hole of the 96 well-plate with five repeats for every rat. Each plate was induced with bovine globulin (ConA) and lipopolysaccharide (LPS), incubated in 5% CO_2_ at 37°C for 48 h, and added to 10 *μ*L of MTT culture solution with further incubation for another 2 h. The proliferation of lymphocytes was detected with dual wavelength at 450 and 650 nm (reference wavelength) using the enzyme labeling instrument. The spleens of all rats were dissected and weighed. The spleen index was calculated as the ratio (mg/g) of spleen wet weight versus body weight.

The article "Antiarthritic Activity of Qi-Wu Rheumatism Granule (a Chinese Herbal Compound) on Complete Freund's Adjuvant-Induced Arthritis in Rats" was retracted in 2026. Reasons: plagiarized images; overlap with other authors' work; unreliable results or conclusions; concerns about the images.

### 2.8. Histology Assay of the Synovial Tissue

At the end of the experiment (day 35), the rats' right hind limbs were dissected and fixed with 10% formaldehyde solution for 48 h. The tissues were embedded in paraffin and sliced. The sections were stained with hematoxylin and eosin (HE) and evaluated by two trained observers who were blinded to the experimental groups. Histological assessment of joint damage was carried out on the basis of articular cartilage damage, underlying bone destruction, and inflammatory cells infiltrate. The cartilage damage was semiquantified with a Mankin scale [22], with* 0-1* indicating invasion of the tidemark by blood vessels,* 0–4* indicating loss of matrix staining, and* 0–6* indicating cartilage structural compromise, with a maximum score of 12 points. The histological scores on bone destruction and inflammatory cells infiltration were scored on a four-scale:* 3*, severe;* 2*, moderate;* 1*, mild; and* 0*, normal [23]. The mean of three sections per rat was used as independent data for statistical analysis.

## 3. Results

### 3.1. Safety Evaluation of QWRG

Compared with the normal control group, the normal physiological function of the mice following intragastric administration of QWRG remained intact. In particular, there were no obvious abnormalities, toxic reactions, or death occurrence up to 14 days after the treatment. In contrast, in the early growth stage of the mice (before the age of 10 days), the growth in the QWRG group was significantly slower than that in the control group as evidenced by the body weight changes. Subsequently, the trend of the weight change was basically comparable between the two groups. This might indicate that the initial differences were due to the large QWRG dose that may have limited the mice feeding, thus resulting in slower growth at early administration. After 10 days of adaptation, the weight growth was comparable between the two groups (Figure 1), which implied that QWRG had no negative effects on growth. In addition, there were no obvious changes in the location, size, color, and adhesion of the organs and no abnormal changes such as fluid or tumor in the viscera surfaces and sections. Taken together, these results confirmed that a large QWRG dose (40 mL/kg) had no acute toxic effects and no influence on the growth of mice, thus implying its safety.

The article "Antiarthritic Activity of Qi-Wu Rheumatism Granule (a Chinese Herbal Compound) on Complete Freund's Adjuvant-Induced Arthritis in Rats" was retracted in 2026. Reasons: plagiarized images; overlap with other authors' work; unreliable results or conclusions; concerns about the images.

### 3.2. The Role of QWRG in the Treatment of AIA Rats

#### 3.2.1. Effects of QWRG on the Paw Swelling

The paw swelling of the AIA group significantly increased compared with the control group (*P* < 0.01) and gradually increased after the model manipulation, indicating that the AIA model was established successfully. After administration of QWRG (1.0, 2.0, and 4.0 g/kg), the paw swelling volume was significantly reduced in the treated rats compared with the AIA group (*P* < 0.05 or *P* < 0.01); this reduction was less pronounced than that of the DEX group (*P* < 0.01; Table 1). The above results show that the QWRG has obviously relieved RA paw swelling, even though still significantly weaker than DEX.

#### 3.2.2. Effect of QWRG on the Body Weights

In the AIA group, the rats' body weights gradually decreased and became significantly different compared to the control group starting from treatment day 7 (*P* < 0.05 or *P* < 0.01). In the rats treated with QWRG (2.0 and 4.0 g/kg), the body weights were significantly different throughout the treatment compared with the AIA group (*P* < 0.05 or *P* < 0.01, resp.), but not with the DEX group (Table 2).

#### 3.2.3. Effect of QWRG on the Arthritic Score

The morphological variation materialized by the arthritic score was significant in all animals of the AIA group (*P* < 0.01). DEX and QWRG (2.0 and 4.0 g/kg) effectively protected the animals against the exaggeration of morphological variation observed in the untreated animals; this was reflected by a significant variation of the arthritic scores between the treated and untreated rats (Table 3).

#### 3.2.4. Effect of QWRG on the Mechanical Nociceptive Threshold

After the administration of QWRG (2.0 and 4.0 g/kg), a significant protective effect against the mechanical pain was observed compared with the AIA group (*P* < 0.05 or *P* < 0.01). However, there was little improvement observed in the mechanical withdrawal threshold in the group treated with low-dose QWRG (1.0 g/kg). DEX showed significant improvement in the mechanical withdrawal threshold between day 1 and day 35 (*P* < 0.05 or *P* < 0.01), which was more pronounced than that induced by QWRG (Table 4). These results showed that QWRG has significantly relieved the mechanical nociceptive threshold.

The article "Antiarthritic Activity of Qi-Wu Rheumatism Granule (a Chinese Herbal Compound) on Complete Freund's Adjuvant-Induced Arthritis in Rats" was retracted in 2026. Reasons: plagiarized images; overlap with other authors' work; unreliable results or conclusions; concerns about the images.

### 3.3. The Impact of QWRG on Serum Biochemical Indicators and Immune Indicators

#### 3.3.1. Effects of QWRG on Serum RF, MDA, ALP, AST, and ALT

Based on Table 5, the serum levels of RF, MDA, ALP, AST, and ALT significantly increased in the AIA group compared with the control group (*P* < 0.01). In animals treated with higher QWRG doses (2.0 and 4.0 g/kg) or DEX, all biochemical parameters evaluated tended to return to normal values (*P* < 0.05 or *P* < 0.01, resp.). Nevertheless, the low-dose QWRG (1.0 g/kg) had nearly no effect on the biochemical indexes (*P* > 0.05), and the effects of high-dose QWRG (4.0 g/kg) basically equaled those of DEX (*P* < 0.05; Table 5).

#### 3.3.2. Effects of QWRG on Serum IL-1*β*, TNF-*α*, IL-16, and IL-2

The inflammatory cytokines IL-1*β*, TNF-*α*, IL-16, and IL-2 of the AIA group were significantly higher than those of the controls (*P* < 0.01). The positive control groups (DEX) and QWRG (2.0 and 4.0 g/kg) displayed all significantly reduced IL-1*β*, TNF-*α*, IL-16, and IL-2 levels compared with the AIA group (*P* < 0.05 or *P* < 0.01), and both QWRG doses (2.0 g/kg and 4.0 g/kg) did not differ significantly. However, the 2.0 g/kg QWRG dose induced significantly weaker effects than the DEX treatment (*P* < 0.05). All these results indicated that QWRG enhanced the immune function in rats, regulated the secretion of inflammatory cytokines, and improved the inflammatory symptoms of RA (Table 6).

#### 3.3.3. Effect of QWRG on the Spleen Index and Spleen Lymphocyte Proliferation

Due to the inflammatory stimulation by adjuvant, the spleen index and T lymphocyte proliferation rate were increased in the AIA group (*P* < 0.01); DEX and QWRG (2.0 and 4.0 g/kg) obviously reduced the spleen index and the proliferation rate of T lymphocytes compared with the AIA group (*P* < 0.05 or *P* < 0.01), while treatment with 2.0 g/kg QWRG resulted in significantly weaker effects than the DEX treatment (*P* < 0.05). These results showed that QWRG can inhibit the ConA- and LPS-induced proliferation of lymphocytes in the spleen (Table 7).

### 3.4. Pathological Changes of the Synovial Membrane following QWRG Treatment

Typical microphotographs of knee joints sections stained with HE illustrated the severity of the joint damage, and histological analyses were performed to investigate whether QWRG relieved the histological changes in knee joint of the AIA rats (Figure 2). In the normal group, the articular cavity was clearly visible, and there was no pathological change in the synovium. The synovial layer was composed of synovial cells and orderly arranged with no inflammatory cell infiltration and a smooth articular cartilage surface. The pathological slides of the AIA group showed matrix thickening, subsynovial collagen fiber structural changes, inflammatory cell infiltration, and obvious capillary hyperplasia. Compared with the AIA rats, QWRG (2.0 and 4.0 g/kg) and DEX ameliorated the above-mentioned pathological changes to varying degrees. Mankin semiquantified analysis of the knee joint sections further indicated that QWRG effectively reduced the cartilage damage (Figure 3(a)), with statistical significance at the higher doses (2.0 and 4.0 g/kg; *P* < 0.01). In addition, accompanied with the relief of cartilage damage, the severity of the underlying bone destruction and inflammatory cells infiltration was also attenuated by QWRG in a dose-dependent manner (*P* < 0.05 or *P* < 0.01; Figures 3(b) and 3(c)).

The article "Antiarthritic Activity of Qi-Wu Rheumatism Granule (a Chinese Herbal Compound) on Complete Freund's Adjuvant-Induced Arthritis in Rats" was retracted in 2026. Reasons: plagiarized images; overlap with other authors' work; unreliable results or conclusions; concerns about the images.

### 3.5. Immunohistochemical Changes of IL-1*β*, TNF-*α*, and IL-16 in Synovium

The IL-1*β*, TNF-*α*, and IL-16 positive cells were found distributed throughout the synovium, especially in the synovial sublining regions (Figures 4(a), 5(a), and 6(a)). Compared with the control group, the expression of IL-1*β*, TNF-*α*, and IL-16 in the AIA group was significantly enhanced (*P* < 0.01). In addition, compared with the AIA group, there was a significant reduction in the expression of IL-1*β*, TNF-*α*, and IL-16 in rats treated with 2.0 g/kg and 4.0 g/kg QWRG and DEX-treated rats (*P* < 0.05 or *P* < 0.01). Furthermore, the efficacy of QWRG treatment at of 4.0 g/kg was similar to that of DEX treatment (*P* > 0.05), while the 2.0 g/kg QWRG dose exerted weaker effects than the DEX treatment (*P* < 0.05; Figures 4(b), 5(b), and 6(b)). These results suggested that QWRG could significantly reduce the expression of IL-1*β*, TNF-*α*, and IL-16 in the synovium of AIA rats.

## 4. Discussion

Rheumatoid, with symptoms such as swelling, release of RF (autoantibody), deformity, and systemic change, is an autoimmune disease characterized by chronic inflammation of the synovial joint. In RA, swelling of the synovium due to the proliferation of synovial cells is the main actor in the cartilage deterioration [24]. Bone erosion, associated with increased and prolonged inflammation, affects 80% of patients and occurs rapidly [25]. In addition, the imbalance of the immune function mainly reflects the imbalance between cellular immunity and humoral immunity. Cellular immunity relatively increases and Th1 cells become activated, thus leading to the secretion of proinflammatory cytokines, while the humoral immunity decreases, and the Th2 inflammatory cytokines secretion decreases [26]. Studies showed that the cytokines produced from mononuclear macrophages and lymphocytes in the synovium play an important role in the pathogenesis of RA [27, 28]. Furthermore, the complex role of the cytokine networks is a key factor in the persistence of RA lesions and the progression of the disease [29]. In the TCM theory, the RA-related symptoms belong to the category of Bi Zheng, which can be manifested as arthralgia and dyskinesia of the joints and dampness and heat of the limbs. QWRG is a TCM compound, and it can dispel cold and relieve pain. In this study, from the evaluation of the safety experiment, the oral administration of 40 mL/kg QWRG did not induce any toxicity in normal mice and did not affect growth, suggesting that the administration of QWRG at this clinical dose would be safe and would not ensue any adverse effects in mice in the context of RA treatment.

The article "Antiarthritic Activity of Qi-Wu Rheumatism Granule (a Chinese Herbal Compound) on Complete Freund's Adjuvant-Induced Arthritis in Rats" was retracted in 2026. Reasons: plagiarized images; overlap with other authors' work; unreliable results or conclusions; concerns about the images.

The AIA rats are an experimental model of RA that shares many pathological features with RA including extremities swelling, synovial hyperplasia, proliferation of synovial tissue, destruction of cartilage, and excessive inflammation. After the AIA rat model was successfully established, we explored the antiarthritic effect of different QWRG doses in the AIA rats. Our results indicated that QWRG (2.0 and 4.0 g/kg) had obviously relieved the AIA paw swelling (Table 1), while the change in body weight was significant throughout the treatment (Table 2), although to a lesser extent it was compared with the DEX treatment. In addition, the QWRG treatment could significantly alleviate the variation of arthritic scores (Table 3) and improve the mechanical nociceptive threshold in the AIA rats (Table 4). These results suggested that QWRG possesses obvious anti-inflammation effects, though with a lesser efficacy than DEX. Previous studies have indicated that TCMs are effective for RA, including* Nux vomica*,* Tripterygium wilfordii*, and orientvine in treating RA [30–33]. In terms of the mechanisms, several TCMs primarily inhibit the expression of cytokines associated with RA to exert their anti-RA effects [34, 35].

To evaluate the antiarthritic property of a drug, the levels of RF, MDA, ALP, AST, and ALT provide an excellent and simple tool. In the present study, the activities of these biomarkers significantly increased in the AIA rats [36]. These enzymes, when released into the circulation during the bone formation and resorption, will be involved in localized bone loss such as bone erosion and periarticular osteopenia [37]. In this study, the levels of AST and ALT were decreased in rats treated with QWRG. This result implies that QWRG can relieve the liver toxicity induced by AIA. In addition, with the QWRG treatments, the increased levels of serum RF, MDA, and ALP were also significantly attenuated (Table 5), indicating that QWRG is effective on AIA.

The article "Antiarthritic Activity of Qi-Wu Rheumatism Granule (a Chinese Herbal Compound) on Complete Freund's Adjuvant-Induced Arthritis in Rats" was retracted in 2026. Reasons: plagiarized images; overlap with other authors' work; unreliable results or conclusions; concerns about the images.

The histological examination and analysis of the knee joint damage were measured by HE staining (Figure 2). Mankin scores were calculated to assess the severity of the cartilage damage. The results suggested that QWRG effectively reduced the severity of cartilage damage in the AIA rats, with statistically significant effects at 2.0 and 4.0 g/kg QWRG (Figure 3(a)). In addition, the severity of the underlying bone destruction and inflammatory cells infiltration was also attenuated by QWRG in a dose-dependent manner (Figures 3(b) and 3(c)), suggesting that QWRG significantly relieved the inflammation of the synovium and improved the cartilage in the AIA rats, even though still significantly weaker than DEX.

In RA, the cytokines can be divided into two categories according to their different sources. One is produced by T lymphocytes, and the other is mainly produced by monocytes/macrophages, including IL-1, TNF, IL-5, IL-18, IL-15, IL-6, IL-12, and IL-17. A variety of factors are interdependent and their interaction results in a large network of cytokines, which restrict or promote the occurrence and development of various diseases. For example, IL-1*β* is an important factor in the development of RA pathology, which can be detected in the joint cavity, and it can assist cell migration and stimulate endothelial cells. Therefore, inhibiting the production of IL-1*β* is one approach for treating RA. As “sister cell cytokines” of IL-1, the effective TNF-*α* target cells and their functions are also very similar. The high expression of TNF-*α* in RA can cause local joint tissue destruction and clinical symptoms [38]. The overexpression of TNF-*α* could result in severe arthritis in mice, while the pharmacological inhibition of the TNF-*α* activity can significantly improve the clinical symptoms of RA [39]. Furthermore, IL-16 is another proinflammatory cytokine secreted by T lymphocytes. In RA, IL-16 can not only destroy the cartilage collagen but also stimulate the differentiation of osteoclast and inhibit the bone synthesis [40]. In addition, IL-16 can also play a synergistic role with TNF-*α* and IL-1*β* to amplify the inflammatory response [41]. This present study focused on investigating the lymphocytes and inflammatory cytokines in AIA rats in addition to exploring the pharmacodynamics of QWRG for a preliminarily inquiry of the cellular and molecular mechanisms of QWRG on relieving AIA. In accordance with the histologic and immunochemical results, QWRG (2.0 and 4.0 g/kg) can significantly alleviate the inflammation of the synovial cavity in RA rats and reduce the grading of synovitis through inhibiting the expressions of IL-1*β*, TNF-*α*, and IL-16 in the serum and synovium of RA rats. It can also antagonize the proliferation of lymphocytes induced by ConA and LPS and the spleen index in rats. The present results indicated that the anti-RA effect of QWRG is profound and that its underlying mechanism might be associated with decreasing the release of cytokines, regulating the function of the spleen, and elevating the immunologic function.

The article "Antiarthritic Activity of Qi-Wu Rheumatism Granule (a Chinese Herbal Compound) on Complete Freund's Adjuvant-Induced Arthritis in Rats" was retracted in 2026. Reasons: plagiarized images; overlap with other authors' work; unreliable results or conclusions; concerns about the images.

In conclusion, our study revealed that QWRG effectively inhibited inflammation and cartilage damage in AIA rats. Taken together with the preventive effects on cartilage damage and relatively lower adverse effects, it is reasonable to regard QWRG as a potential antiarthritic drug. However, further work is still needed to identify the detailed mechanisms underlying this effect. Our findings present some experimental evidence that the reduction of IL-1*β*, TNF-*α*, and IL-16 in the serum and synovial tissue and the reduction of lymphocyte proliferation might be of potential clinical interest in RA treatment. Thus, in the light of the above-mentioned findings, it could be asserted that QWRG could serve as a promising herbal drug that will open a new window for the treatment of RA.

## Figures and Tables

**Figure 1:** Effects of QWRG on normal mice weight (animals received intragastric administrating with QWRG during 14 d; the values of weight are means, with their standard errors represented by vertical bars. Herein, circle and squares represented the QWRG treatment group and control, resp.).

**Figure 2:** Effect of QWRG on synovium damage of rats with AIA (representative histopathologic photos of knee joint sections from different groups with H&E staining, taken from control rats, AIA model rats, QWRG-treated rats of 1.0 g/kg, 2.0 g/kg, and 4.0 g/kg, and DEX-treated group).

**Figure 3:** Semiquantified analysis of the protective effect of QWRG on synovium damage. (a) Mankin scores on cartilage damage; (b) histological scores on underlying bone destruction; (c) histological scores on inflammatory cells infiltration. Tissues from three different rats in each group and 10 randomly selected areas from each slide were analyzed. Data are mean ± SD (*n* = 10). ^*∗∗*^*P* < 0.01 versus control; compared with AIA group, when *P* is less than 0.01 or 0.05, it means very significant difference, designated by ## or #; ^&^*P* < 0.05 versus DEX.

**Figure 4:** Immunohistochemical results of IL-1*β* in synovium (immunohistochemistry of IL-1*β* in the knee joints taken from control rats, AIA model rats, QWRG-treated rats of 1.0 g/kg, 2.0 g/kg, and 4.0 g/kg, and DEX-treated group. Magnification ×200. Tissues from three different rats in each group and 10 randomly selected areas from each slide were analyzed. Quantitative data (mean ± SD) are presented using the average density values of the IL-1*β* positive regions. ^*∗∗*^*P* < 0.01 versus control; ^##^*P* < 0.01 versus AIA group; ^&^*P* < 0.05 versus DEX).

The article "Antiarthritic Activity of Qi-Wu Rheumatism Granule (a Chinese Herbal Compound) on Complete Freund's Adjuvant-Induced Arthritis in Rats" was retracted in 2026. Reasons: plagiarized images; overlap with other authors' work; unreliable results or conclusions; concerns about the images.

**Figure 5:** Immunohistochemical results of TNF-*α* in synovium (immunohistochemistry of TNF-*α* in the knee joints taken from control rats, AIA model rats, QWRG-treated rats of 1.0 g/kg, 2.0 g/kg, and 4.0 g/kg, and DEX-treated group. Magnification ×200. Tissues from three different rats in each group and 10 randomly selected areas from each slide were analyzed. Quantitative data (mean ± SD) are presented using the average density values of the TNF-*α* positive regions. ^*∗∗*^*P* < 0.01 versus control; ^#^*P* < 0.05, ^##^*P* < 0.01 versus AIA group; ^&^*P* < 0.05 versus DEX).

**Figure 6:** Immunohistochemical results of IL-16 in synovium (immunohistochemistry of IL-16 in the knee joints taken from control rats, AIA model rats, QWRG-treated rats of 1.0 g/kg, 2.0 g/kg, and 4.0 g/kg, and DEX-treated group. Magnification ×200. Tissues from three different rats in each group and 10 randomly selected areas from each slide were analyzed. Quantitative data (mean ± SD) (*n* = 10) are presented using the average density values of the IL-16 positive regions. ^*∗∗*^*P* < 0.01 versus control; ^##^*P* < 0.01 versus AIA group; ^&^*P* < 0.05 versus DEX).

**Table 1:** Effects of QWRG in AIA model on paw swelling ($\overset{-}{x}\pm s$, *n* = 10).

Groups	Paw swelling (mL)					
	0 d	7 d	14 d	21 d	28 d	35 d
Control	0.03 ± 0.02	0.03 ± 0.12	0.09 ± 0.07	0.03 ± 0.11	0.04 ± 0.12	0.04 ± 0.16
AIA group	1.58 ± 0.41^*∗∗*^	2.15 ± 0.40^*∗∗*^	2.71 ± 0.66^*∗∗*^	2.93 ± 0.77^*∗∗*^	2.94 ± 0.73^*∗∗*^	3.32 ± 1.26^*∗∗*^
DEX (5 mg/kg)	1.49 ± 0.20	0.53 ± 0.43^##^	0.64 ± 0.24^##^	0.86 ± 0.32^##^	0.78 ± 0.32^##^	0.90 ± 0.57^##^
QWRG						
1.0 g/kg	1.64 ± 0.52	1.68 ± 0.55^#&&^	2.25 ± 0.37^#&&^	2.31 ± 0.12^#&&^	2.37 ± 0.49^#&&^	2.44 ± 1.18^#&&^
2.0 g/kg	1.64 ± 0.42	1.76 ± 0.48^#&&^	2.17 ± 0.49^#&&^	2.13 ± 0.28^#&&^	2.14 ± 0.88^#&&^	2.06 ± 0.13^#&&^
4.0 g/kg	1.62 ± 0.71	1.12 ± 0.58^##&&^	1.53 ± 0.22^##&&^	1.29 ± 0.736^##&&^	1.20 ± 0.75^##&&^	1.26 ± 0.94^##&&^

The values from 10 different rats in each group. Data are mean ± SD. ^*∗∗*^*P* < 0.01 versus control; ^#^*P* < 0.05, ^##^*P* < 0.01 versus model; ^&&^*P* < 0.01 versus DEX.

**Table 2:** Effects of QWRG in AIA model on relative body weight ($\overset{-}{x}\pm s$, *n* = 10).

Groups	Relative body weight (%)					
	0 d	7 d	14 d	21 d	28 d	35 d
Control	100.0	101.4 ± 12.2	102.3 ± 12.6	104.6 ± 12.1	106.5 ± 11.9	109.1 ± 10.2
AIA group	100.0	96.5 ± 10.3	94.2 ± 9.6^*∗*^	93.8 ± 9.6^*∗∗*^	92.0 ± 10.2^*∗∗*^	92.5 ± 11.6^*∗∗*^
DEX (5 mg/kg)	100.0	99.2 ± 11.3	98.3 ± 9.4	99.2 ± 9.2^#^	98.8 ± 10.5^#^	100.5 ± 9.7^#^
QWRG						
1.0 g/kg	100.0	97.1 ± 10.2	96.1 ± 10.6	95.2 ± 10.8^&^	94.5 ± 10.9^&^	94.7 ± 9.4^&^
2.0 g/kg	100.0	98.3 ± 9.9	97.1 ± 10.1	97.3 ± 9.8^#^	96.8 ± 9.8^#^	96.1 ± 10.2^#&^
4.0 g/kg	100.0	99.2 ± 11.3	99.1 ± 9.4^#^	98.1 ± 9.7^#^	97.3 ± 8.9^##^	98.5 ± 9.7^##^

The values from 10 different rats in each group. Data are mean ± SD. ^*∗*^*P* < 0.05, ^*∗∗*^*P* < 0.01 versus control; ^#^*P* < 0.05, ^##^*P* < 0.01 versus model; ^&^*P* < 0.05 versus DEX.

The article "Antiarthritic Activity of Qi-Wu Rheumatism Granule (a Chinese Herbal Compound) on Complete Freund's Adjuvant-Induced Arthritis in Rats" was retracted in 2026. Reasons: plagiarized images; overlap with other authors' work; unreliable results or conclusions; concerns about the images.

**Table 3:** Effects of QWRG in AIA model on arthritic score ($\overset{-}{x}\pm s$, *n* = 10).

Groups	Arthritic score					
	0 d	7 d	14 d	21 d	28 d	35 d
Control	0	0	0	0	0	0
AIA group	4.3 ± 0.8^*∗∗*^	5.3 ± 0.3^*∗∗*^	8.2 ± 0.6^*∗∗*^	7.4 ± 0.6^*∗∗*^	7.0 ± 0.9^*∗∗*^	7.1 ± 11.6^*∗∗*^
DEX (5 mg/kg)	4.1 ± 0.9	4.2 ± 0.8^#^	2.3 ± 0.4^##^	2.2 ± 0.2^##^	1.8 ± 0.5^##^	1.5 ± 0.7^##^
QWRG						
1.0 g/kg	4.0 ± 0.6	5.1 ± 0.7	7.8 ± 0.6	7.4 ± 0.8	7.1 ± 0.4	6.9 ± 0.6
2.0 g/kg	4.2 ± 0.5	4.8 ± 0.4^&^	6.8 ± 0.9^#&&^	6.3 ± 0.5^#&&^	6.0 ± 0.8^#&&^	6.1 ± 0.5^#&&^
4.0 g/kg	4.3 ± 0.8	4.3 ± 0.1^#^	3.4 ± 0.7^##^	3.1 ± 0.5^##^	2.9 ± 0.8^##^	3.0 ± 0.4^##^

The values from 10 different rats in each group. Data are mean ± SD. ^*∗∗*^*P* < 0.01 versus control; ^#^*P* < 0.05, ^##^*P* < 0.01 versus model; ^&^*P* < 0.05, ^&&^*P* < 0.01 versus DEX.

**Table 4:** Effects of QWRG in AIA model on mechanical nociceptive threshold ($\overset{-}{x}\pm s$, *n* = 10).

Groups	Paw withdrawal latency (%)					
	0 d	7 d	14 d	21 d	28 d	35 d
Control	100.0	99.2 ± 3.5	99.4 ± 5.5	98.7 ± 4.2	97.6 ± 3.4	99.1 ± 6.2
AIA group	100.0	35.4 ± 5.3^*∗∗*^	33.6 ± 7.6^*∗∗*^	32.4 ± 5.5^*∗∗*^	32.0 ± 6.2^*∗∗*^	30.1 ± 4.8^*∗∗*^
DEX (5 mg/kg)	100.0	44.4 ± 6.9^#^	52.7 ± 6.8^##^	63.5 ± 9.1^##^	65.8 ± 8.5^##^	72.3 ± 11.7^##^
QWRG						
1.0 g/kg	100.0	35.4 ± 5.7	36.3 ± 9.6	37.4 ± 7.6	36.8 ± 6.8	37.1 ± 8.2
2.0 g/kg	100.0	37.7 ± 6.8	42.8 ± 7.8^##&^	52.9 ± 9.2^##&^	51.5 ± 6.9^##&^	53.6 ± 8.1^##&^
4.0 g/kg	100.0	41.4 ± 6.4^#^	45.5 ± 6.4^##^	58.8 ± 7.3^##^	60.2 ± 8.15^##^	60.1 ± 5.9^##^

The values from 10 different rats in each group. Data are mean ± SD. ^*∗∗*^*P* < 0.01 versus control; ^#^*P* < 0.05, ^##^*P* < 0.01 versus model; ^&^*P* < 0.05 versus DEX.

**Table 5:** Effects of QWRG in AIA model on serum biochemical indicators ($\overset{-}{x}\pm s$, *n* = 10).

Groups	RF (IU/mL)	MDA (nmol/mL)	ALP (U/L)	AST (U/L)	ALT (U/L)
Control	—	3.8 ± 0.6	80.4 ± 4.2	42.4 ± 2.0	45.7 ± 5.3
AIA group	87.4 ± 2.4^*∗∗*^	7.1 ± 1.4^*∗∗*^	483.2 ± 29.0^*∗∗*^	142.3 ± 9.5^*∗∗*^	172.6 ± 9.2^*∗∗*^
DEX (5 mg/kg)	35.5 ± 1.9^##^	4.6 ± 0.6^##^	178.4 ± 16.9^##^	78.9 ± 5.9^##^	99.3 ± 8.1^##^
QWRG					
1.0 g/kg	81.8 ± 3.0	7.0 ± 2.1	455.3 ± 23.2	142.0 ± 11.2	168.6 ± 8.4
2.0 g/kg	46.9 ± 3.2^##&^	6.2 ± 1.5^#&^	345.5 ± 12.3^##&&^	112.3 ± 8.4^&^	143.3 ± 9.5^#&^
4.0 g/kg	37.9 ± 4.1^##^	4.9 ± 2.2^##^	248.0 ± 22.6^##^	89.3 ± 7.8^##^	111.4 ± 10.4^##^

The values from 10 different rats in each group. Data are mean ± SD. ^*∗∗*^*P* < 0.01 versus control; ^#^*P* < 0.05, ^##^*P* < 0.01 versus AIA group; ^&^*P* < 0.05, ^&&^*P* < 0.01 versus DEX.

The article "Antiarthritic Activity of Qi-Wu Rheumatism Granule (a Chinese Herbal Compound) on Complete Freund's Adjuvant-Induced Arthritis in Rats" was retracted in 2026. Reasons: plagiarized images; overlap with other authors' work; unreliable results or conclusions; concerns about the images.

**Table 6:** Effects of QWRG in AIA model on serum immune indicators ($\overset{-}{x}\pm s$, *n* = 10).

Groups	IL-1*β* (pg/mL)	TNF-*α* (pg/mL)	IL-16 (pg/mL)	IL-2 (pg/mL)
Control	215.3 ± 58.5	402.4 ± 73.19	10.2 ± 0.6	85.3 ± 8.3
AIA group	451.9 ± 37.5^*∗∗*^	825.9 ± 61.15^*∗∗*^	28.4 ± 1.6^*∗∗*^	163.4 ± 9.0^*∗∗*^
DEX (5 mg/kg)	328.4 ± 33.9^##^	591.6 ± 81.42^##^	13.4 ± 1.6^##^	96.7 ± 6.8^##^
QWRG				
1.0 g/kg	429.6 ± 47.5	818.8 ± 114.42	25.9 ± 2.2	158.5 ± 5.9
2.0 g/kg	373.4 ± 49.3^##&^	702.5 ± 94.11^##&^	17.2 ± 1.9^##&^	108.6 ± 6.0^##&^
4.0 g/kg	342.5 ± 61.1^##^	618.6 ± 91.06^##^	12.4 ± 2.3^##^	90.5 ± 4.9^##^

The values from 10 different rats in each group. Data are mean ± SD. ^*∗∗*^*P* < 0.01 versus control; ^##^*P* < 0.01 versus AIA group; ^&^*P* < 0.05 versus DEX.

**Table 7:** Effects of QWRG in AIA model on spleen index and spleen lymphocyte proliferation ($\overset{-}{x}\pm s$, *n* = 10).

Groups	Spleen index	OD_450_	
		ConA	LPS
Control	3.8 ± 0.5	402.43 ± 73.2	10.2 ± 0.6
AIA group	5.9 ± 0.7^*∗∗*^	825.88 ± 61.2^*∗∗*^	28.4 ± 1.6^*∗∗*^
DEX (5 mg/kg)	4.4 ± 0.9^##^	591.6 ± 81.4^##^	13.4 ± 1.6^##^
QWRG			
1.0 g/kg	5.6 ± 0.5	818.82 ± 114.4	25.9 ± 2.2
2.0 g/kg	5.0 ± 0.6^&^	702.53 ± 94.1^#&^	17.2 ± 1.9^##&^
4.0 g/kg	4.5 ± 1.1^##^	618.58 ± 91.6^##^	12.4 ± 2.3^##^

The values from 10 different rats in each group. Data are mean ± SD. ^*∗∗*^*P* < 0.01 versus control; ^#^*P* < 0.05, ^##^*P* < 0.01 versus AIA group; ^&^*P* < 0.05 versus DEX.
